# *In Silico* design of a multi-epitope vaccine for Human Parechovirus: Integrating immunoinformatics and computational techniques

**DOI:** 10.1371/journal.pone.0302120

**Published:** 2024-12-04

**Authors:** Arnob Sarker, Md. Mahmudur Rahman, Chadni Khatun, Chandan Barai, Narayan Roy, Md. Abdul Aziz, Md. Omar Faruqe, Md. Tofazzal Hossain

**Affiliations:** 1 Department of Biochemistry and Molecular Biology, University of Rajshahi, Rajshahi, Bangladesh; 2 Bioinformatics and Structural Biology Lab, Department of Biochemistry and Molecular Biology, University of Rajshahi, Rajshahi, Bangladesh; 3 Department of Computer Science and Engineering, University of Rajshahi, Rajshahi, Bangladesh; University of Chittagong, BANGLADESH

## Abstract

Human parechovirus (HPeV) is widely recognized as a severe viral infection affecting infants and neonates. Belonging to the *Picornaviridae* family, HPeV is categorized into 19 distinct genotypes. Among them, HPeV-1 is the most prevalent genotype, primarily associated with respiratory and digestive symptoms. Considering HPeV’s role as a leading cause of life-threatening viral infections in infants and the lack of effective antiviral therapies, our focus centered on developing two multi-epitope vaccines, namely HPeV-Vax-1 and HPeV-Vax-2, using advanced immunoinformatic techniques. Multi-epitope vaccines have the advantage of protecting against various virus strains and may be preferable to live attenuated vaccines. Using the NCBI database, three viral protein sequences (VP0, VP1, and VP3) from six HPeV strains were collected to construct consensus protein sequences. Then the antigenicity, toxicity, allergenicity, and stability were analyzed after discovering T-cell and linear B-cell epitopes from the protein sequences. The fundamental structures of the vaccines were produced by fusing the selected epitopes with appropriate linkers and adjuvants. Comprehensive physicochemical, antigenic, allergic assays, and disulfide engineering demonstrated the effectiveness of the vaccines. Further refinement of secondary and tertiary models for both vaccines revealed promising interactions with toll-like receptor 4 (TLR4) in molecular docking, further confirmed by molecular dynamics simulation. *In silico* immunological modeling was employed to assess the vaccine’s capacity to stimulate an immune reaction. *In silico* immunological simulations were employed to evaluate the vaccines’ ability to trigger an immune response. Codon optimization and *in silico* cloning analyses showed that *Escherichia coli (E*. *coli)* was most likely the host for the candidate vaccines. Our findings suggest that these multi-epitope vaccines could be the potential HPeV vaccines and are recommended for further wet-lab investigation.

## 1. Introduction

Human parechovirus (HPeV) is a non-enveloped, positive-sense, single-stranded RNA virus that belongs to the Picornaviridae family and the Parechovirus genus. The virus genome is approximately 7.4 kilobases in length and contains a single open reading frame encoding a polyprotein which cleaved into structural and nonstructural proteins. The genome structure is similar to other picornaviruses, with an internal ribosome entry site for translation. The structural proteins, which form the viral capsid, are encoded in the P1 region of the polyprotein and include VP0, VP1, and VP3 and nonstructural proteins in the P2 and P3 regions. The viral capsid comprises 60 protomer units with VP0, VP1, and VP3, with VP1 containing the receptor-binding domain which mediates attachment to host cells [1, 2]. Currently, HPeV is categorized into 19 genotypes based on distinct VP1 sequences. Among them, the majority of available data pertain to genotypes 1–8, with HPeV1 and HPeV3 being the most prevalent strains [3, 4]. HPeVs are the second most common cause of viral meningitis in children. The majority of these infections occur in newborns under 90 days of age which may lead to severe neurodevelopmental consequences, including encephalitis, meningitis, myocarditis, and sepsis [5].

Particularly in underdeveloped nations, there is a lack of comprehensive data on incidence of parechovirus infections. A research conducted on healthy children in the Philippines revealed that 24.7% of the children had enteroviruses, which includes parechovirus [6]. Its prevalence was also found to be between 27 to 80% in an Indian study on acute viral hepatitis, indicating the significant prevalence in underdeveloped nations. High parechovirus prevalence is also reported in industrialized nations; this may be because of subclinical infections or cross-reactivity. Immunocompromised people and pregnant women are more vulnerable to it with death rates ranging from 1- 4% [7]. An analysis of canine parvovirus enteritis in Nigeria demonstrates the importance of host specificity in virus epidemiology, with a much lower prevalence of 7.97% [2]. Therefore, based on available data, human HPeV is a major public health concern, particularly in underdeveloped nations where prevalence rates range from 24.7% to 80%.

While pocapavir might be considered for emergency use, obstacles exist in the current HPeV vaccination methods. Like SARS-CoV-2, rapid evolution of virus affects the efficacy of vaccinations. The HPeV vaccine’s development is complicated by its increased age group and unusual adverse effects. To understand immunity and develop new vaccines, pathogen complexity, and evolution must be taken into consideration. A comprehensive strategy incorporating virus evolution, flexible populations, and cutting-edge genomic technologies for vaccine development is required to overcome these obstacles [8, 9].

In these phenomena, Immunoinformatics is being employed to address this challenge, enabling more effective vaccine design through a precise, rapid, and efficient method of vaccine creation. By employing appropriate immunoinformatics techniques, it is possible to create multi-epitope vaccines [10]. Multi-epitope vaccines offer several advantages in vaccine development. They can trigger robust and diverse immune responses, as seen in the development of multi-epitope vaccines against HPV16, Nipah virus, Brucella, influenza, and Vibrio spp. These vaccines utilize immunoinformatics to predict epitopes for cytotoxic T lymphocytes (CTLs), helper T lymphocytes (HTLs), and B cells, enhancing the vaccine’s immunogenicity. Multi-epitope vaccines can induce specific CD4 and CD8 T cell expansion, elevate cytokine levels, and promote memory T cell proliferation, leading to potent immune responses against various pathogens. Additionally, these vaccines can provide long-lasting protection, reduce the risk of vaccine escape mutants, and offer practicality in terms of manufacturing and genetic manipulability, making them promising candidates for future vaccine development [11–16]. Thus, a multi-epitope vaccine for HPeV may hold potential, and an immunoinformatic study to explore this possibility may help identify alternative approaches to vaccine development for entire the global population.

Thus in this study, we conducted immunoinformatic analyses to design two multi-epitope vaccines (HPeV-Vax-1 and HPeV-Vax-2) against HPeV. In order to construct consensus sequences, we compiled the three viral protein (VP0, VP1, and VP3) sequences of six HPeV strains. After identifying T-cell and linear B-cell epitopes, we assessed the protein antigenicity, toxicity, allergenicity, and stability of these sequences. The epitopes were then fused together with the proper adjuvants and linkers to create the basic structures of the vaccine. The development and refinement of these two vaccines were further carried out in secondary and tertiary models. Molecular docking of both vaccine models revealed promising interactions with toll-like receptor 4 (TLR4), supported further by dynamics simulation. The capability of the vaccine to provoke an immune response was evaluated through computational immunological modeling.

## 2. Materials and methods

### 2.1. Retrieval and identification of protein sequences

Though HPeV have several strains, consensus sequences for each viral protein were first constructed. To build consensus sequences, the fasta format of six strains (Q66578.1, O73556.1, BAC23086.1, ABC41566.1, Q9YID8.1, and BAF63403.1) were derived from the dataset available on NCBI (https://www.ncbi.nlm.nih.gov/). Next, using Seaview software, consensus sequences for the three viral proteins (VP0, VP1, and VP1) from each of these six strains were constructed by aligning their fasta formats [17]. The antigenicity of three consensus sequences was evaluated by utilizing the VaxiJen v2.0 server for prediction. (http://www.ddg-pharmfac.net/vaxijen/VaxiJen/VaxiJen.html) [18].

### 2.2. MHC-І binding (Cytotoxic T Lymphocyte (CTL)) epitopes prediction

CTLs are one type of immune cell that can kill other cells. CTLs identify and eliminate virus-infected cells through their recognition and targeted killing mechanism. CTLs can identify peptides originating from viral antigens that are attached to MHC proteins on the cell surface [19]. So, predicting T-cell-inducing peptide responses is an essential stage in the development (https://services.healthtech.dtu.dk/services/NetCTL-1.2/) was utilized to predict 9-mer CTL epitopes for the specified proteins [20]. It predicts CTL epitopes by combining predictions of proteasomal cleavage, TAP transport efficiency, and MHC class I binding affinity. Each of the three proteins was screened for CTL epitopes which are capable of recognized by 12 MHC class I supertypes. The threshold for epitope prediction was defined as 0.75, indicating that only epitopes scoring equal to or higher than this value were considered significant for further analysis. The predicted CTL epitopes underwent additional scrutiny to assess their antigenicity using Vaxijen v2.0, toxicity utilizing ToxinPred server (https://webs.iiitd.edu.in/raghava/toxinpred/design.php) [21] and potential to induce allergies through AllerTOPv2.0 server (https://www.ddg-pharmfac.net/AllerTOP/index.html) [22]. ToxinPred server utilizes support vector machine (SVM) method because of its ability to distinguish toxic epitopes from non-toxic ones.

### 2.3. MHC-ІІ binding (Helper T Lymphocyte (HTL) epitopes prediction

The presence of virus-specific CD4+ T cells (HTLs) is essential for inducing both cellular and humoral immunity during viral infections. Therefore, it is proven that HTL epitopes will serve as a crucial element in the formulation and effectiveness of immunotherapeutic vaccines. [23, 24]. The chosen proteins underwent prediction of 15-mer HTL epitopes utilizing the NetMHCII v2.3 server, which can be accessed at (https://services.healthtech.dtu.dk/services/NetMHCII-2.3/). The NetMHCII tool predicts peptide binding affinities to MHC-II molecules [25]. The investigation involved scanning each of the three proteins to identify HTL epitopes that could be recognized by different alleles of HLA-DP, HLA-DR, and HLA-DQ. The cutoff points distinguishing between strong and weak binders were established at 2% and 10%, respectively. Following the prediction process, the HTL epitopes underwent analysis for antigenicity, toxicity, and allergenicity. Furthermore, for assessing their capability to trigger IFN-γ and IL-4 inducing T-helper cells, the epitopes ranked highest were forwarded to the IFNepitope server (http://crdd.osdd.net/raghava/ifnepitope/) [26] and the IL4pred server (http://crdd.osdd.net/raghava/il4pred/) [27] correspondingly.

### 2.4. Linear B-cell epitope prediction

Upon antigen recognition, B cells differentiate with the assistance of CD4+ T follicular helper (TFH) cells, resulting in the generation of plasma cells that secrete antibodies and memory B cells capable of neutralizing and impeding virus entry [28]. Linear B-cell epitopes were predicted using the IEDB tool, accessible at (http://tools.iedb.org/bcell/) [29] and using Bepipred Linear Epitope Prediction 2.0 method. This method utilizes the combination of hidden Markov model with one of the best propensity scale methods. Finally, the predicted B epitopes underwent for evaluation like other epitopes.

### 2.5. Population coverage analysis

Human leukocyte antigens (HLA) frequencies show widespread variation across human populations and geographic location [30]. Population coverage analysis plays a critical role in vaccine development, ensuring the ability to bind to various alleles of HLA supertypes. The population coverage tool provided by IEDB, accessible at (http://tools.iedb.org/population/) was utilized to estimate the extent of coverage provided by the selected epitopes within the specified target population [31]. In our population coverage analysis, we evaluated the HLA binding alleles associated with the selected MHC class-II epitopes. Nine different geographical regions along with world population were chosen for this analysis.

### 2.6. Multi-epitope vaccines development

Two multi-epitope vaccines were formulated by organizing chosen CTL, HTL, and linear B-cell epitopes with appropriate linkers and adjuvants. Adjuvants are vaccine components that enhance the potency, range, and durability of the immune response [32]. We selected the adjuvant, 50S ribosomal protein L7/L12 (Locus RL7_MYCTU), identified by its UniProt ID P9WHE3 [33] and a 6x His tag [34] to construct one vaccine. Adjuvant (Human β-defensin-3 sequence (UniProt id. Q5U7J2)) and a 11 aa (amino acid) TAT sequence tag were used to construct the other vaccine [35]. The first step involved adding an adjuvant to the N-terminal of the vaccine, which is facilitated by the EAAAK linker. To augment the vaccine’s immunogenicity, we inserted the pan-HLA DR binding epitope (PADRE epitope, 13 aa) after the linker [36]. Afterward, the CTL epitopes were interconnected through the AAY linker, while the HTL epitopes were joined via the GPGPG linker, and the B-cell epitopes were connected using the KK linker. For epitope class separation, a GGGS linker was introduced [34]. Linkers play a crucial role in effectively separating individual epitopes and facilitating the construction of a more stable protein structure [37]. Finally, the tags were incorporated into the vaccine’s C-terminal for further purification assays.

### 2.7. Vaccine evaluation: Antigenicity, allergenicity, solubility, and physicochemical profile

Allergenicity prediction for the two constructed vaccines was conducted using both the AllerTOP v.2.0 and AllergenFP v.1.0 [38] servers. Furthermore, the antigenicity assessment of the designed vaccines was conducted through comprehensive analysis using the http://scratch.proteomics.ics.uci.edu/. The assessment of vaccine solubility was performed with thorough analysis employing both Protein-Sol [39] and SOLpro [40] servers. The Expasy ProtParam server was employed to calculate various physicochemical properties of vaccine constructs e.g. formula, number of atoms, molecular weight, extinction coefficient, grand average of hydropathicity (GRAVY), instability index, theoretical isoelectric point (pI), aliphatic index, and half-life. (https://web.expasy.org/protparam/) [41]. The Deep TMHMM tool (http://www.cbs.dtu.dk/services/TMHMM/) was employed to predict the number of transmembrane (TM) helices within the proposed vaccine [42].

### 2.8. Prediction of secondary structure

Utilizing the NetSurfP-3.0 server, accessible at (https://services.healthtech.dtu.dk/services/NetSurfP-3.0/) we performed predictions on the secondary structure characteristics, encompassing α-helices, β-sheets, and random coils, of the constructed vaccines. This server employs the ESM-1b language model to encode the proteins, followed by analysis with a deep neural network [43].

### 2.9. Prediction of tertiary structure, refinement, and validation

The 3D tertiary structure prediction of the multi-epitope vaccines was conducted using the I-TASSER server (https://zhanggroup.org/I-TASSER/). The server rearranges amino acid sequences from templates, calculating a C-score to assess the accuracy of the predicted models. In the typical range of -5 to 2, the C-score provides insight into model quality, where values greater than -1.5 generally signify a correct fold [44, 45].

To enhance the quality of the structure both locally and globally, the GalaxyRefine server (https://galaxy.seoklab.org/cgi-bin/submit.cgi?type=REFINE) was utilized to refine those 3D models of two vaccines [46]. Evaluation of both the initial and tertiary 3D structure was compared through the SWISS-MODEL Structure Assessment (https://swissmodel.expasy.org/assess) [47] and ProSA-web server (https://prosa.services.came.sbg.ac.at/prosa.php) [48]. The Ramachandran plot, derived from SWISS-MODEL [49] visually represents the acceptable and unacceptable dihedral angles (psi—ψ and phi—ϕ) of amino acids, accounting for the side chain’s Van der Waals radius [50]. The server generates a z-score for each query protein, indicating the quality of the protein structures.

### 2.10. Prediction of discontinuous B-Cell epitope

Discontinuous or conformational B-cell epitopes, resulting from protein folding, bring distant residues together to generate them, constituting more than 90% of B-cell epitopes. The revised 3D model of the vaccines underwent analysis using the ElliPro server available at (http://tools.iedb.org/ellipro/) to identify discontinuous B-cell epitopes [51]. This method predicts epitopes by evaluating solvent accessibility and flexibility. Based on the predicted three-dimensional (3D) structure the ElliPro prediction tool identifies antigenic residues

### 2.11. Molecular docking analysis

Molecular docking experiments were conducted using the ClusPro 2.0 server, accessible at (https://cluspro.org/login.php) [52, 53], where a lower energy score indicates better binding affinity. The server executes three computational steps: (i) it performs rigid-body docking by exploring billions of conformations; (ii) it conducts root-mean-square deviation (RMSD)-based clustering of the 1,000 lowest-energy structures to identify the largest clusters that represent the most probable models of the complex; and (iii) it refines the chosen structures through energy minimization. It can handle the maximum grid size of approximately 40 × 10^6^ Å^3^, equivalent to a cube with dimensions of around 350 Å on each side. The initial step involved retrieving the 3D structure of TLR4, specified by its PDB ID (4G8A). Subsequently, preprocessing steps e.g. hetatms and the ligand elimination within TLR4 structure was performed using the Discovery Studio software [54]. Following this, the 3D model of the two refined multi-epitope vaccines and TLR4 were docked using the server, with the former designated as ligands and the latter as the receptor. The binding free energy was determined through the application of the subsequent equation:

$$E=0.40E_{rep}+-0.40E_{att}+600E_{elec}+1.00E_{DARS}$$

[52, 55]. Finally, PDBsum (http://www.ebi.ac.uk/thornton-srv/databases/pdbsum/) [56] and PyMOL software [57] was used to visualize the interactions between the vaccines and TLR-4 complexes.

### 2.12 Disulfide engineering of the multi-epitope vaccines

The disulfide engineering of the vaccines were conducted to analyze the conformational stability of folded proteins, utilizing Disulfide by Design 2 server version 2.13 (http://cptweb.cpt.wayne.edu/DbD2/) [58]. All the parameters were kept at default including χ3 angle which was set at -87° or +97° and Cα-Cβ-Sγ angle which was set at 114.6° ± 10. Residue pairs with energy levels below 2.2 Kcal/mol were selected and modified to cysteine residues to create disulfide bridges [59]. The disulfide bonds were chosen using a criteria of 2.2 Kcal/mol since 90% of native disulfide bonds have an energy value of less than that [58].

### 2.13. Molecular Dynamics Simulation (MDS) of vaccine TLR4 complexes

We conducted MD simulations using YASARA software [60] and the AMBER14 [61] force field to explore the stability and molecular mobility of the docked vaccine-TLR complexes. At first, the hydrogen bonding network of the complexes was refined and submerged in a TIP3P water model prior to running the simulation. [62]. The solvent density was adjusted to 0.997 g/ml to maintain periodic boundary conditions during the simulation. Each simulation was initially subjected to energy minimization using the steepest descent algorithm for 5000 cycles. Each simulation was conducted under typical physiological conditions (298 K temperature, pH 7.4, 0.9% NaCl) [63] and employed a multiple time-step algorithm [64] which involved 2.50 femtoseconds (fs) time-step interval. A molecular dynamics simulation of 100 ns was carried out using a Berendsen thermostat [65] to regulate the temperature, while maintaining constant pressure throughout the simulation. These conditions helped establish a stable and realistic environment for the simulation. The YASARA [66] macro’s default script and the SciDAVis (https://scidavis.sourceforge.net/) were used to conduct the primary analysis. Simulation trajectories were recorded at regular intervals of 250 picoseconds (ps). Various graphs, such as RMSD, radius of gyration (Rg), RMSF, H-bond, and PCA, were analyzed to check the flexibility and stability of the complexes.

### 2.14. *In silico* immune simulation

Using the online immune response simulation program C-ImmSim, it is feasible to predict the profiles of both cell-mediated and humoral immune responses in mammals subsequent to vaccination [67], accessible at https://kraken.iac.rm.cnr.it/C-IMMSIM. To predict immunological interactions, C-ImmSim uses a matrix-based strategy and machine learning techniques based on the principle of agent-based modelling [67]. All parameters were maintained at their default settings, with the exception of the time step. The vaccines were injected with time step at 1, 84, 170 where each time step equal to 8 hours [68]. Three injections were given at intervals of four weeks during the simulations.

### 2.15 Codon optimization and *in silico* cloning analysis

Methods to efficiently express the protein in the host organism are the final stage in vaccine creation. The goal of this *in silico* cloning method was to predict the dynamics of expression of protein. As the host organism, *Escherichia coli* K12 was used to produce a codon-optimized nucleic acid sequence from the vaccine’s amino acid sequence, which was then uploaded to the JCAT server [69]. In order for digestion and cloning of the vaccine model inside the pET-28a (+) vector, the cDNA sequence was examined using SnapGene software to identify possible restriction enzyme cut sites.

## 3. Results

### 3.1 Retrieval and identification of protein sequences

Sequence alignment was conducted using the Muscle tool within the Seaview software. The analysis revealed that though the strains are highly conserved there are few variations among them.

To address this issue, consensus sequences were constructed (**S1–S3 Figs**). The Consensus threshold value was set at 50% and no gaps were allowed during the construction of these sequences. As determined by the VaxiJen v2.0 server, the antigen score for three target proteins was higher than 0.4, which is the specified threshold value. The consensus sequences and corresponding antigenicity scores are given in **Table 1**.

**Table 1:** Consensus sequences of the proteins and their vaxijen scores.

Proteins	Consensus Sequence	Vaxijen score
VP0	METIKSIADMATGTKTIDSTINVNEINGNASGGDILTKVADDASNLGPNCFATTSEPENKDVVQATTTVNTTNLTQHPSAPTMPFTPDFSNVDNFHSMAYDITTGDKNPSKLIRLTWTRQHIHVELPKAFWDQRKPAYGQARYFAAVRCGFHFQVQVNVNQGTAGSALVVYEPKPVVDHKLEFGAFTNLPHVLMNLAETTQADLCIPYVADTNYVKTDSSDLGQLRVYVWTPLSIPSGATNQVDVTVLGSLLQLDFQNPRVYDVDIYDN	0.5515
VP3	PTKRKKKILTMSTKYKWTRNKIDIAEGPGSMNMANVLSTTGAQSVALVGERAFYDPRTAGSKSRFDDLVKIAQLFSVMADSTTPSSSGIDKGYFKWSATPQIVHRNVVLNQFPNLNFVNSYSYFRGSLIIRLSVYASTFNRGRLRMGFFPNTTDTTSELDNAIYTICDIGSDNSFEITIPYSFSTWMRKTNGHPIGLFQIEVLNRLTYNSSSPNEVHCIVQGRLGDAKFFCPTGSLVTFQ	0.5730
VP1	NSWGSQMDLTDPLCIEDDEDCKQTISPNELGLTSAQDDGPLGNEKPNYFLNFRMNVDIFTVSHTKVDNIFGRAWFAHDFNEGTWRQLFPKEGHGLSLLFAYFTGELNIHVLFLSGFLRVAHTYDTNRNFLSSNGVITVPAGEQMTLSVPFYSNKPLRTVRDALGYLMCKPFLTGTTSGKIEVYLSLRCPNFFFPLPAPKPTSRALRGDMANLSDQ	0.4030

### 3.2 MHC-І binding CTL epitopes prediction

A collective count of 591 CTL epitopes from three protein sequences were identified using the NetCTL v1.2 server. To identify the most promising CTL epitopes from a pool of epitopes, emphasis was placed on those epitopes demonstrating robust binding affinity to at least three MHC class I super types. Subsequently, these epitopes underwent filtration based on criteria such as toxicity, antigenicity and allergenicity and finally 8 epitopes were selected for further process (**S1–S3 Tables**).

### 3.3 MHC-ІІ binding HTL epitopes prediction

A cumulative count of 650 HTL epitopes from three protein sequences were identified using the NetMHCII v2.3 server. After that, 500 HTL epitopes were selected from the initial 650 epitopes, based on their affinity (IC50) values being less than 50 nM, as high-binding peptides typically have IC50 values below 50 nM. Among the 500 epitopes, 82 were selected that exhibited strong binding affinity to at least five human MHC class II alleles. Finally, a total of 8 HTL epitopes were selected from these 82 epitopes based on their assessment studies and their capability to induce both IFN-γ and IL-4 (**S4–S6 Tables)**.

### 3.4 Linear B-cell epitope prediction

The IEDB server successfully detected a total of 24 linear B-cell epitopes derived from three protein sequences. Epitopes with a length greater than 10 amino acids were examined for their antigenicity, toxicity, and allergenicity, resulting in the selection of a total of 6 linear B-cell epitopes **(S7–S9 Tables**).

### 3.5 Population coverage analysis

Population coverage analysis of epitope vaccines is a critical step in vaccine development, ensuring that the vaccine can effectively bind to multiple alleles of HLA supertypes. In our study, the selected epitopes provided coverage for 99.4% of the world population (**Fig 1** and **S10 Table**). Furthermore, the epitopes exhibited coverage of 100% in the specific regions that were selected (**S4 Fig**).

**Fig 1:** World population coverage of Class I and Class II combined, as predicted by the IEDB tool, is depicted in bar chart. The chart shows the number of epitope and allele combinations (x-axis) recognized by different regions of the world population. Here approximately 5.75% can be recognized by 26 and 29 combinations. The right-hand y-axis shows the cumulative percent of world population coverage. Cumulatively, adding from right to left, it is expected that at least 18 epitopes can be recognized in 90% of individuals. Similarly, slightly over 80% of the world population would recognize 21 and more, while 60% would recognize 26 and more. The coverage value for the whole group of Class I and Class II epitopes is 99.99%.

### 3.6 Multi-epitope vaccines development

To prevent duplication of epitopes within the vaccine construct, any epitopes with sequences overlapping those of other epitopes were excluded. Three CTLs epitopes, ALVGERAFY, KILTMSTKY and KQTISPNEL were found overlapping in the shortlisted B-cell epitope VLSTTGAQSV**ALVGERAFY**DPRTAGSKSRFD, RKK**KILTMSTKYK**WTRNKIDIAEGPGSMNM, and SQMDLTDPLCIEDDEDC**KQTISPNEL**GLTSAQDDGPLGNEKPNYF, respectively, all from the same protein. To prevent redundancy, these three CTL epitopes were excluded from the final vaccine construction. Finally, two multi-epitope vaccines (**HPeV-Vax-1 and HPeV-Vax-2**) were constructed by fusing the finalized 5 CTL, 8 HTL and 6 B-cell epitopes along with different adjuvants, linkers and tags (**Fig 2, S11, S12 Tables**).

**Fig 2:** Here is a representation of a multi-epitope vaccine. Five CTL epitopes (illustrated in mint), eight HTL epitopes (illustrated in grey), and 6 B-cell epitopes (illustrated in blue) are joined with AAY, GPGPG linkers and KK linkers, respectively. They are separated from each other by GGGS linker (shown in Orange). (A) At the beginning of the sequence, the 50S ribosomal protein L7/L12 (Locus RL7_MYCTU), identified with UniProt ID P9WHE3 (illustrated in orchid), is connected via an EAAAK linker (highlighted in yellow), whereas a 6-histidine tag (depicted in pink) is attached to the sequence’s end for distinction. In (B), the human β-defensin-3 adjuvant with **UniProt ID Q5U7J2** (shown in orchid) and a TAT sequence (11 aa) tag (shown in pink) are used to construct the HPeV-Vax-2 model.

### 3.7 Evaluation of antigenicity, allergenicity, solubility and physicochemical properties of constructed vaccines

Hpev-Vax-1 and 2 have molecular weight (MW) of 61.82 kDa and 53.59 kDa, respectively, while Protein-Sol and SOLpro servers estimated that the vaccines produced are in a soluble form (0.99 for HPeV-Vax-1 and 0.98 for Hpev-Vax2) with theoretical isoelectric points (pI) 9.34 (alkaline) and 9.91 (alkaline) respectively. Therefore, the vaccines are suitable for vaccine application and are easily purifiable (MW < 110 kDa).

A protein is considered stable if its instability index is below 40, whereas a value above 40 suggests that the protein may be unstable [41]. The computed instability index of Hpev-Vax1 (28.00) and Hpev-Vax2 (31.68) indicates that the designed vaccines are considered as stable proteins. Moreover, the aliphatic index of Hpev-Vax1 (69.03) and Hpev-Vax2 (61.88) suggests that they are thermo-stable. In addition, the GRAVY (Grand Average of Hydropathicity) value for a peptide or protein is determined by summing the hydropathy values of all the amino acids in the sequence and then dividing this sum by the total number of residues. Hydropathy values or scales were developed based on the hydrophilic and hydrophobic characteristics of each of the 20 amino acid side chain [70]. The gravy values of the two vaccines Hpev-Vax1 and Hpev-Vax2 were -0.356 and -0.451 which indicate that the vaccines are hydrophilic, thus more soluble in water. The estimated half-life duration of all vaccine constructs is greater than 30 hours in-vitro. In yeast and E. coli (in-vivo), the estimated half-life of all constructs is greater than 20 hours and 10 hours, consecutively. Furthermore, the absence of predicted transmembrane (TM) helices suggests that the vaccines are well-suited for application (**S13 Table**).

### 3.8 Prediction of secondary structure

The secondary structure of HPeV-Vax-1 revealed that the resultant structure consists of 15.544% α -helix, 9.845% β -sheets, and 74.611% random coil. HPeV-Vax-2 similarly exhibits 13.42% α -helix structure, 8.41% β -sheets, and 78.15% random coil (**S5 Fig**).

### 3.9 Prediction of tertiary structure, refinement, and validation of the vaccine construct

Five 3D structures were produced by the I-TASSER server for the two candidate vaccines considering the top ten threading templates, with Z-score covering a range from 1.04 to 5.49. All threading templates exhibited proper alignment, as evidenced by Z-scores greater than 1, and vice versa. The five models of Hpev-vax-1 and Hpev-Vax-2 had C-scores of − 0.83, − 1.25, − 2.77, − 3.16, and − 3.04 and -1.16, -3.11, -2.97, -3.53, -3.54, respectively. We selected the models with C-score of −1.25 and -1.16 (C-score > -1.5 indicates a correct global topology). Then the selected model underwent refinement using the GalaxyRefne server. The server supplied five polished models of the vaccines. Model-4 was deemed the most optimal refined model for Hpev-vax-1, and Model-1 was deemed the best refined model for Hpev-vax-2 based on its quality scores (**S14 Table**). Higher GDT-HA scores are indicative of superior quality models. Notably, both model-4 and model-1 showcased GDT-HA scores of 0.9378 and 0.9078, respectively, surpassing all other refined models. A reduced RMSD value suggests increased stability, and an RMSD value falling between 0 and 1.2 is typically considered acceptable [71]. In this context, the RMSD score for these models are 0.463 and 0.530. The MolProbity score serves as an indicator of the crystallographic resolution attained for the protein’s 3D model, where a decrease in score corresponds to a reduction in critical errors [72]. Model-4 and model-1 had a MolProbity score of 2.554 and 2.624, respectively, significantly lower compared to the initial model. The Clash score reflects the quantity of unfavourable all-atom spatial overlaps, whereas the bad rotamers score denotes the count of residues with limited potential for rotational movement in their side chains [73]. Lower scores for these parameters signify a better 3D structure of the protein. Specifically, model-4’s Clash and poor rotamers scores were 17.6 and 1.5, respectively, while model-1’s scores were 18.0 and 1.5. In the original Hpev-vax1 model, 69.13% of the residues were in the preferred region, according to a Ramachandran plot analysis. However, in the improved model, 84.58% of the residues occupied the same region. Similarly, in the original Hpev-vax2 model, 51.11% of the residues were in the preferred area, compared to 80.08% in the revised model (**S6 and S7 Figs**).

### 3.10 Discontinuous B-Cell epitope prediction

Briefly, seven epitopes were predicted for Hpev-vax1, involving residue sizes ranging from 5 to 141, with scores varying between 0.545 and 0.746. For HPeV-Vax-2, five epitopes were predicted, involving residues sizes ranging from 9 to 95, with scores in the range of 0.552 to 0.774 **(S15, S16 Tables, S8 and S9 Figs)**.

### 3.11 Disulfide engineering of the multi-epitope vaccines

Disulfide by Design 2 server identifies potential sites within a protein structure where amino acid pairs are likely to form disulfide bonds. For this experiment, only pairs with bond energies below 2.2 kcal/mol were selected. In Hpev-vax1, it was found that the bond energy of five amino acid pairs was less than 2.2 kcal/mol: 56 ALA and 98 ASP, 62 GLU and 112 ALA, 114 ASP and 134 LYS, 223 ILE and 297 PHE and finally 421 ASP and 427 ALA. In HPeV-Vax-2: 15 GLY and 80 PHE, 33 CYS and 41 CYS, 314 VAL and 338 PHE (**S10 Fig**).

### 3.12 Molecular docking analysis

Molecular docking experiments were conducted to explore the binding strength between the TLR-4 receptor and designed vaccines. To perform the molecular docking studies, the ClusPro v2.0 server was utilized for docking between the TLR-4 receptor and the vaccine constructs. Twenty-six models were generated for each vaccine. Among them, we selected cluster No. 13 for each vaccine with the largest cluster size of 13 and 17 members and the minimum energy of -1465.8 Kcal/mol and -1595.6 Kcal/mol for vaccine HPeV-Vax-1 and HPeV-Vax-2 respectively. The interaction between TLR-4 receptor and vaccine constructs are visualized in **S11 Fig**. Further interpretations of the involvement interacting amino acids in disulfide and hydrogen bonds, salt bridges, in addition to non-bonded contacts were analyzed using the PDBsum server. In the receptor (TLR4) and ligand (vaccine construct) of HPeV-Vax-1, 31 hydrogen bonds and 6 salt bridges were formed, while in HPeV-Vax-2, 15 hydrogen bonds and 4 salt bridges were identified (**Fig 3, S12 and S13 Figs**). The PRODIGY server was utilized to determine the Gibbs free energy or ΔG value, confirming the binding affinity between the TLR-4 receptor and the two constructed vaccines. The ΔG values of -11.1 kcal/mol, -12.8 kcal/mol, along with dissociation constant (K_d_) values of 7.3E-9, 4.3E-10 for the docked complexes of HPeV-Vax-1 and HPeV-Vax-2, respectively, indicate that the interactions with TLR-4 receptor for both vaccines are energetically appropriate.

**Fig 3:** The interactions between the residues of the both chain A of TLR-4 and vaccine. (A) Map of total interacting residues and bonds between the HPeV-Vax-1 and TLR-4 protein chain A. (B) Map of total interacting residues and bonds between the HPeV-Vax-2 and TLR-4 protein chain A.

### 3.13 Molecular dynamic (MD) simulations of vaccine TLR4 complexes

The docked vaccine (HPeV-Vax-1 and HPeV-Vax-2) with TLR4 complexes were subjected to 100 ns molecular dynamics simulations. The average RMSD values for the Cα backbone of TLR4- HPeV-Vax-1 and TLR4- HPeV-Vax-2 complexes are 3.015 Å and 3.062 Å respectively **(Fig 4A)**. The maximum RMSD values for the TLR4-HPeV-Vax-1 and TLR4-HPeV-Vax-2 complexes were 4.422Å and 4.269Å, respectively. Despite this, both complexes showed almost similar pattern and remained stable during the time period except some minor fluctuation between 65 to 75 ns. Moreover the radius of gyration (Rg) analysis revealed that TLR4-HPeV-Vax-1 had a slightly higher average Rg value than TLR4-HPeV-Vax-2, with values of 41.015Å and 40.785 Å, respectively **(Fig 4B)**. In addition, both complexes remained relatively stable throughout the entire simulation. To determine whether the TLR-vaccine complexes affect the dynamic behavior of residues, the RMSF values of the vaccine complex were compiled (**Fig 4C)**. Both complexes showed some fluctuations in the range of 555–645 and 1110–1500 residues from 3.5 to 8 Å and 3.5 to 6.2 Å respectively. However the overall RMSF for both of the complexes were below 3 Å. We evaluated the intermolecular hydrogen bonding in the TLR4-vaccine complexes during the entire simulation period. Intermolecular hydrogen bonds play a key role in maintaining protein stability, with a higher number of H-bonds indicating greater stability of the complex. The number of hydrogen bonds in both complexes remained relatively high and stable, ranging from 1025 to 1150 throughout the entire simulation (**Fig 4D**). We analyzed the PCA values for the TLR 3-vaccine and TLR 9-vaccine complexes throughout the simulation. These calculations were crucial in assessing the stability of each complex, as lower distribution of PCA values indicates higher stability. From **Fig 4E and 4F**, it can be seen that both of the complexes exhibited some conformational changes due to its distribution. From the above analysis it can be clearly interpreted that all the complexes were structurally stable.

**Fig 4:** 100 ns MD simulation of the TLR4 and vaccine complexes. (A) Root mean square daviation (RMSD) plot and (B) Radius of gyration (Rg) plot. (C) Root mean square fluctuation (RMSF) plot (D) Time evolution of intra-molecular hydrogen bonds (E) PCA analysis of HPeV-Vax-1 and (F) PCA analysis of HPeV-Vax-2.

### 3.14 *In silico* immune simulation

The *in silico* simulation of the humoral and cell-mediated immune responses of two constructed vaccines (HPeV-Vax-1 and HPeV-Vax-2) was carried out using the C-ImmSim web server **(Figs 5 & 6)**. From the figures, it can be seen that both candidate vaccines exhibited comparable patterns in terms of immune cell induction. The HPeV-Vax-2 vaccine exhibits slightly stronger IgM and IgG antibody responses after the 2^nd^ and 3^rd^ injections compared to HPeV-Vax-1 **(Figs 5A and 6A**). On the other hand, HPeV-Vax-1 produces the slightly more active B cell and Th cell than HPeV-Vax-2 following the 2^nd^ and 3^rd^ injections. Overall, population of memory cells (B and T cell) is the main disparity between the first injection and the subsequent ones for both vaccines (**Figs 5B–5D and 6B–6D**). Moreover, **Figs 5E, 5F and 6E, 6F** ensure the involvement of innate (i.e., macrophage) and cytokine based immune response. Therefore, following the injection, significant levels of IL-2 and interferon-gamma are produced [72]. So, these two vaccine candidates have the ability to stimulate positive immunological responses.

**Fig 5:** *In silico* immune simulation of vaccine HPeV-Vax-1 includes the following components. (A) Antibodies generated in response to antigen injections were depicted as various colored peaks, while the antigen itself was represented in black (B) B cell population (C,D) Active T-helper (TH) cell population and Active T-cytotoxic (TC) cell populations. The resting state indicated cells that had not been exposed to the antigen (vaccine). In contrast, the anergic state showed T-cells’ tolerance to the antigen as a result of repeated exposures. (E) Macrophage population; (F) The secretion of induced cytokines and the diversity measurement of IL-2 levels.

**Fig 6:** *In silico* immune simulation of vaccine **HPeV-Vax-2** includes the following components- (A) Antibodies generated in response to antigen injections were depicted as various colored peaks, while the antigen itself was represented in black (B) B cell population (C,D) Active T-helper (TH) cell population and Active T-cytotoxic (TC) cell populations. The resting state indicated cells that had not been exposed to the antigen (vaccine). In contrast, the anergic state showed T-cells’ tolerance to the antigen as a result of repeated exposures. (E) Macrophage population; (F) The secretion of induced cytokines and the diversity measurement of IL-2 levels.

### 3.15 Codon optimization and *In Silico* cloning analysis

The JCat server-generated two optimized cDNA sequences from the amino acid sequences of our constructed vaccines (HPeV-Vax-1 and HPeV-Vax-2), demonstrating favorable parameters. The Codon Adaptation Index (CAI) values for HPeV-Vax-1 and HPeV-Vax-2 were 0.544 and 0.604, respectively, suggesting a high likelihood of increased expression. The GC content values for both vaccines are 68.45% and 68.003% respectively, which fall in the optimal range of 30–70%. The multi-epitope vaccine insert is carried in the expression vector pET 28a (+) **(Fig 7)**.

**Fig 7:** *In silico* cloning of the **(A)** HPeV-Vax-1 vaccine and **(B)** HPeV-Vax-2 vaccine construct into pET-28a (+) vector. The inserted segment is indicated in red.

## 4. Discussion

Human Parechovirus (HPeV) primarily affects newborns and infants, potentially causing a broad spectrum of clinical symptoms, including severe encephalitis that can lead to paralysis, making it imperative to prevent this potential life-threatening disease [74]. Emerging HPeV infections demand the development of new therapeutic strategies. Epitope-based vaccines offer a promising approach to designing effective vaccines that are highly potent, logistically feasible, and offer improved safety. By eliminating unfavorable epitopes that can cause detrimental immune responses, multi-epitope vaccines have a capacity to elicit particular immunogenic responses based on conserved epitopes throughout entire antigenic sequences. [75]. As of now, there is no specific vaccine available as the primary preventive measure to prevent HPeV infection [76]. The goal of this study was to generate novel multi-epitope HPeV vaccine constructions that could stimulate immune responses in infected persons by using immunoinformatics techniques. Three outer membrane proteins (VP0, VP1, and VP3) from six HPeV strains (HPeV-1 to HPeV-6) were aligned to construct a consensus protein sequence. These consensus sequences then underwent different types of assessment based on the criteria such as antigenicity, allergenicity and toxicity. Following this several suitable T-cell and B-cell epitopes were identified from the protein sequences. These discovered epitopes are essential to adaptive immunity; MHC-II epitopes support humoral and cellular immune responses, whereas MHC-I epitopes fight viruses and infected cells [77]. Population coverage of the epitopes were found significant with 99.99% worldwide. This was also supported by other studies [78]. Two separate adjuvant peptide sequences and various combinations of immune enhancers were utilized to connect specific epitopes in order to create two vaccine constructions [32].

These multi-epitope structures were shown to be non-allergic and non-toxic, further highlighting their potential as vaccine candidates. The vaccines showed the potential antigenicity with a score of 0.70 (**S13 Table**). However, GRAVY value of HPeV-Vax-1 and HPeV-Vax-2 were estimated -0.356 and -0.451 along with the solubility score of 0.99 and 0.98 respectively, which means the vaccines are hydrophilic in nature and easily soluble in water [79, 80]. This vaccines were also examined for potential disulfide bond-forming amino acid pairs to create the mutant variant. Five amino acid pairings for HPeV-Vax-1 and three amino acid pairing for HPeV-Vax-2 that satisfied the selection criterion of bond energies less than 2.2 kcal/mol which is required for mutant protein generation. These pairs included 56 ALA and 98 ASP, 62 GLU and 112 ALA, 114 ASP and 134 LYS, 223 ILE and 297 PHE, 421 ASP and 427 ALA for HPeV-Vax-1 and 15 GLY and 80 PHE, 33 CYS and 41 CYS, 314 VAL and 338 PHE for HPeV-Vax-2. Disulfide engineering found beneficial for vaccine design in other studies [81].

Understanding how antigens interact with receptor molecules is essential for developing vaccines. This requires structural knowledge. Predicting and optimizing the three-dimensional architectures of the two vaccine designs guaranteed structural stability. Moreover TLR-4 immune cell receptor, which is essential for immune cell activation and innate immunity, exhibited substantial binding affinities with the vaccination designs, according to molecular docking studies. In our study we found that, HPeV-Vax-1 and HPeV-Vax-2 displayed lowest amount of energy of -1465.8 Kcal/mol and -1595.6 Kcal/mol when interacting with TLR-4 receptor. Additionally, the docked complexes of HPeV-Vax-1 and HPeV-Vax-2 had ΔG values of -11.1 kcal/mol, -12.8 kcal/mol respectively, and indicating appropriate interaction with TLR-4 receptor. Several studies also suggested that lower energy provides better interaction [82, 83]. Furthermore, molecular dynamics simulations confirmed the robust interactions of the two vaccines with the TLR-4 receptor, securing molecular stability within a cellular environment. In this study we found that average RMSD value of the TLR4- HPeV-Vax-1 and TLR4- HPeV-Vax-2 complexes were 4.422Å and 4.269Å along with Rg value of 41.015 Å and 40.785 Å, respectively. Lower RMSD and Rg value were also suggested as better result in many studies [82, 84]. Thus, it proves the stability of our vaccine complexes. The RMSF analysis revealed the variation of atoms from their average positions, allowing us to assess the flexibility of different regions within the complex. Hydrogen bonding refers to the calculation of total hydrogen bonds, encompassing those formed within the peptide or between the peptide and the surrounding solvent. These bonds are tracked based on the distance and angle between the donor and acceptor atoms. The TLR4-vaccine complexes exhibited a higher number of hydrogen bonds, suggesting greater stability. PCA measures the fluctuations in the number of amino acid residues, where smaller fluctuations indicate a more stable and compact protein structure. Thus, the complexes appear to be more stable due to lower fluctuations [85].

The outcomes of the immune simulation were similar to those of natural cellular immunogenic responses, with increased levels of immune components and the establishment of B- and T-cell memory after vaccination. This implies the potential for a variety of immunogenic reactions. Our vaccines were able to generate good amount of antibodies, B cell, T cell, macrophage and diverse amount of cytokines and IL2 populations which confirms a potential immunogenic response in human body after vaccine injection [86]. To confirm the efficacy of the developed vaccine, serological analysis is essential, and the *E*. *coli* expression system is regarded as well-suited for the cloning and production of recombinant peptides, facilitating the validation process. The Codon Adaptation Index (CAI) values for HPeV-Vax-1 and HPeV-Vax-2 were 0.544 and 0.604 and GC content were 68.45% and 68.003% respectively, which indicates good expression of vaccines inside *E*.*coli*. This is also supported by other studies [87]. These findings suggest the potential for stable immunogenic responses.

*In silico* immune simulations are valuable and can guide laboratory experiments, thereby saving time and resources [88]. The next phase comprises preclinical trials to validate the study’s findings and evaluate the immunogenicity of the developed vaccine, as well as immunological assays to validate the results. Some studies also suggested the importance of *in vivo* and *in vitro* analysis for further validations [89, 90]. Moreover, further *in vivo* and *in vitro* investigation on expression vectors for vaccine cloning need to be done which might be essential for large scale productivity of the constructed vaccines.

## 5. Conclusion

Human Parechovirus (HPeV) is now widely recognized as a severe viral infection in infants and neonates. Considering HPeV’s significant role as a leading cause of life-threatening viral infections in babies and the lack of effective antiviral therapies, our focus has been on developing two multi-epitope vaccines against HPeV, employing cutting-edge immunoinformatic techniques. To construct these vaccines, we predicted and meticulously screened CTL, HTL, and B-cell epitopes of viral proteins sequentially. The resulting vaccines exhibited all desirable physicochemical features, including solubility, high antigenicity, and a lack of allergenicity.

Through molecular docking analysis, we established the vaccine’s high binding affinity to TLR4. Additionally, using MD simulation, we were able to validate the vaccine’s stability. Immunological simulations confirmed the vaccine’s capability to stimulate the immune system effectively. Furthermore, acceptable Codon Adaptation Index (CAI) and GC content values from codon optimization supported the vaccine’s viability for expression in a bacterial host. Even though this study’s suggested vaccinations are predicated on *in silico* prediction, more research is necessary.

## Supporting information

S1 Table Results of CTL epitope prediction of VP0 protein from Human Parechovirus (HPeV). (DOCX)

S2 Table Results of CTL epitope prediction of VP1 protein from Human Parechovirus (HPeV). (DOCX)

S3 Table Results of CTL epitope prediction of VP3 protein from Human Parechovirus (HPeV). (DOCX)

S4 Table Results of HTL epitope prediction of VP0 protein from Human Parechovirus (HPeV). (DOCX)

S5 Table Results of HTL epitope prediction of VP1 protein from Human Parechovirus (HPeV). (DOCX)

S6 Table Results of HTL epitope prediction of VP3 protein from Human Parechovirus (HPeV). (DOCX)

S7 Table Results of linear B-cell epitope prediction of VP0 protein from Human Parechovirus (HPeV). (DOCX)

S8 Table Results of linear B-cell epitope prediction of VP1 protein from Human Parechovirus (HPeV). (DOCX)

S9 Table Results of linear B-cell epitope prediction of VP3 protein from Human Parechovirus (HPeV). (DOCX)

S10 Table Population coverage table. (DOCX)

S11 Table Final epitopes of vaccine construct. (DOCX)

S12 Table Sequence and vaxijen score of two vaccines. (DOCX)

S13 Table Psychochemical properties of constructed vaccines. (DOCX)

S14 Table Tertiary structure evaluation of constructed vaccines before and after refinement. The selected model has been shown in bold.
(DOCX)

S15 Table Conformation of discontinuous B-cell epitopes in refined vaccines (HPev-Vax-1). (DOCX)

S16 Table Conformation of discontinuous B-cell epitopes in refined vaccines (HPev-Vax-2). (DOCX)

S1 Fig Consensus sequence of protein VP0 from six parechovirus strains. (DOCX)

S2 Fig Consensus sequence of protein VP1. (DOCX)

S3 Fig Consensus sequence of protein VP3. (DOCX)

S4 Fig Regional population Class I and Class II combined coverage as predicted by the IEDB tool (Plot A to H). (DOCX)

S5 Fig Secondary structure evaluation of constructed vaccines. (DOCX)

S6 Fig 3D model construction and validation of HPeV-Vax-1. (DOCX)

S7 Fig 3D model construction and validation of HPeV-Vax-2. (DOCX)

S8 Fig Conformational B-cell epitopes prediction in HPeV-Vax-1. (DOCX)

S9 Fig Conformational B-cell epitopes prediction in HPeV-Vax-2. (DOCX)

S10 Fig The **(A)** original and **(B)** mutant HPeV-Vax-1 and HPeV-Vax-2 before and after disulfide engineering has been shown side by side.
(DOCX)

S11 Fig Docking analysis between TLR-4 receptor and constructed vaccines. (DOCX)

S12 Fig The interactions between the residues of HPeV-Vax-1 and chain B, C of TLR-4. (DOCX)

S13 Fig The interactions between the residues of HPeV-Vax-2 and chain B, C of TLR-4. (DOCX)
